RETRACTED

# High-Quality Nursing Combined with the Whole-Course Responsibility Nursing Intervention Reduces the Incidence of Complications in Severe Aneurysmal Subarachnoid Hemorrhage

**DOI:** 10.1155/2022/3252718

**Published:** 2022-07-16

**Authors:** Xiaoli Qian, Lin Gong, Fen Zhou, Yan Zhang, Haibo Wang

**Affiliations:** ^1^Department of Critical Care Medicine, Hai'an People's Hospital, Nantong, Jiangsu 226600, China; ^2^Neurosurgery Department, Chinese Medical Hospital of Wujin, Wujin, Changzhou, China

## Abstract

**Objective:**

The aim of this study is to study the influence of whole-course responsibility nursing combined with high-quality nursing intervention on the level of life and complications of severe aneurysmal subarachnoid hemorrhage patients with postoperative coma.

**Methods:**

From December 2018 to December 2020, 90 severe aneurysmal subarachnoid hemorrhage patients with postoperative coma were selected and were divided into two groups, the experimental group and the control group, with 45 cases in each group. The control group adopted conventional nursing care, and the experimental group received whole-course responsibility nursing combined with high-quality nursing intervention. The nursing effect, degree of coma, coma recovery, and incidence of complications between all groups were compared.

**Results:**

Compared with the control group, the experimental group yielded more favorable achievement in terms of the nursing effect (*P* < 0.05). Superior levels of the Glasgow Coma Scale (GCS) score, Coma Recovery Scale-Revised (CRS-R) score, GQOLI-74 score, and BI score of the experimental group were obtained and compared with the control group (all *P* < 0.05). The experimental group witnessed a lower complication rate, as compared to the other group (*P* < 0.05).

**Conclusion:**

The whole-course responsibility nursing combined with high-quality nursing intervention is applied to severe aneurysmal subarachnoid hemorrhage patients with postoperative coma, which can substantially optimize the nursing efficiency, improve the degree of coma, help recover consciousness, ameliorate the mental state and the quality of life, and reduce the incidence of complications, which is worthy of clinical application.

## 1. Introduction

Aneurysmal subarachnoid hemorrhage (SAH), as a neurosurgery emergency and severe disease, poses a serious threat to human health with a very high disability rate and mortality rate. In a systematic evaluation and meta-analysis, the overall crude global incidence of aneurysmal SAH across all study periods was 7.9/100,000 person-years [1]. This disease occurs in elderly people, and its morbidity is also witnessing a gradual rise among young people. Surgical treatment is the mainstay for treating severe aneurysmal subarachnoid hemorrhage, but postoperative coma is rather frequent. The failure of regaining consciousness in time will increase the risk of disability and mortality [2–4]. Clinically, there are many causes of spontaneous subarachnoid hemorrhage, the most common being intracranial aneurysm rupture and arteriovenous malformation accounting for 57%, followed by hypertensive intracerebral hemorrhage [5]. However, after some patients died, the cause could not be found at autopsy, and it may be the rupture of aneurysm small arteriovenous malformation to form a thrombus without leaving traces [6]. Furthermore, most autopsies do not examine the venous system or the spinal subarachnoid space, both of which are causes of hemorrhage [7].

RETRACTED

In recent years, the challenge of how to shorten the duration of coma after severe aneurysmal subarachnoid hemorrhage has become a hot research topic. Relevant studies have shown that through external stimulation, the excitability of the patient's cerebral cortex can be enhanced, so that the function of the patient's damaged nerve cells can be restored and the state of consciousness can be improved, thus achieving the purpose of recovery. Patient's consciousness. The Total Responsible Care model further improves the quality of care by dividing nursing responsibilities and stratifying care according to the actual situation of the patient on the basis of the conventional nursing model. In addition, high-quality nursing interventions are an emerging nursing concept. The effective combination of society, psychology, and biology promotes the transformation of the nursing model and its clinical application is remarkable [8, 9]. In this study, we aim to explore the impact of whole-course responsibility nursing combined with high-quality nursing intervention on the level of life and related complications of severe aneurysmal subarachnoid hemorrhage patients with postoperative coma. The report is as follows.

## 2. Materials and Methods

### 2.1. General Information

Ninety patients with severe aneurysmal subarachnoid hemorrhage in postoperative coma who underwent treatment at our hospital from December 2018 to December 2020 were recruited and divided equally into two groups using the random number table method, the experimental group and the control group, with 45 cases in each group. The experiment was approved by the ethics committee.

### 2.2. Inclusion Criteria

The inclusion criteria were as follows: (1) diagnosis of severe aneurysmal subarachnoid hemorrhage [10]; (2) patients aged 18 to 70 years; (3) postoperative coma; and (4) patients and their families voluntarily signed an informed consent form after learning to be informed.

RETRACTED

### 2.3. Exclusion Criteria

The exclusion criteria were as follows: (1) combined liver or renal failure; (2) combined cardiovascular disease; (3) combined ischemic stroke; (4) combined severe infection; and (5) pregnant or lactating women.

### 2.4. Methods

The control group adopted routine nursing intervention. Medical staff should carry out routine perioperative care, provide medication guidance and dietary guidance, ensure a comfortable and clean hospitalization environment, and conduct psychological interventions.

The experimental group adopted whole-course responsibility nursing combined with high-quality nursing intervention. The whole-course responsibility nursing model first required nursing grouping, so that the nursing staff could divide the labor, to carry out the nursing service more smoothly, and ensure a better quality of nursing. Meanwhile, it was necessary to optimize the hospital's traditional nursing model so that the whole-course responsibility nursing model was able to be fully applied and integrated into the nursing work. The nursing work must be carried out systematically and comprehensively, and the sense of responsibility of nursing staff must be enhanced [11–13]. Professional knowledge training for nursing staff was regularly carried out, to effectively improve nursing level of the nursing staff, cultivate the comprehensive level of the nursing staff, and ensure the proficiency and high-level professional skills of the nursing staff in the clinical nursing process. Moreover, it is also crucial to strengthen the professional training, focus on cultivating the risk awareness of nurses, lecture nursing risk cases to nurses, and organize medical staff to learn about risk prevention, which guarantees the calmness and expertness of the nursing staff in risk events, minimizes the damage caused by the risk events, and further improves their professional skills [14–16]. Medical staff needed to perform tactile and auditory wake-up interventions on the patients: according to the principle of “top to down and front to back,” medical staff should appropriately stimulate the patients to wake-up their senses of touch, 30 minutes for 2 times. Because of actual condition of cases, medical staff should develop a targeted auditory wake-up plan for patients, including calling the patients' names beside the bed and reading books to the patients, 40 minutes for each time, once in the morning and once in the evening. Medical staff should also encourage the patients' family members to accompany the patients throughout the entire process and share interesting things with patients, to arouse their memories. By calling the patient's name, a stimulus can be formed to provide the patient with information coding, which in turn stimulates the human body's reflex mechanism, helps the patient regain memory traces, and promotes a membrane potential to generate action potentials [17].

RETRACTED

### 2.5. Observation Indicators

The “Glasgow Coma Scale” [18] (GCS) was used to evaluate the degree of coma of the two groups of patients. The scale mainly includes language response, limb response, and eye-opening response. The higher the score, the less severe the patient's coma.

The “Coma Recovery Scale-Revised” [19] (CRS-R) can evaluate the state of consciousness of all groups of cases; the score was directly proportional to the state of consciousness of the patients.

The nursing influence of all groups of cases was observed. When patient's clinical symptoms were significantly improved, the nursing effect was regarded as markedly effective; when the clinical symptoms improved, the nursing effect was effective; when the clinical symptoms were not improved, the nursing effect was determined as ineffective.

The “General Quality of Life Inventory-74” (GQOLI-74) was used to assess level of life of the all patients between the intervention. The scale includes 4 aspects including psychological, physical, social function, and material life status; all scores are 100 points, the higher score, the better level of life of the patient.

The “Barthel index (BI) Rating Scale” [20] was used to evaluate ability of daily living of patients. The higher score, the better ability of daily living of subjects.

The complication rate of all groups of cases was compared. Complication rate = number of people with complications/total number of people in this group × 100%.

### 2.6. Statistical Analysis

SPSS20.0 was selected to process data in study, and GraphPad Prism 7 (San Diego, USA) was used to draw data. Using *χ*^2^-tests, *t*-test, and normality test, *P* < 0.05 was considered to be significant.

## 3. Results

### 3.1. General Information Comparison

There were no differences in smoking, drinking, and place of residence between all groups of patients (*P* > 0.05), as shown in Table 1.

### 3.2. Comparison of GCS Scores between the Two Groups

A higher level of GCS score was obtained in the experimental group (*P* < 0.05). See Table 2.

### 3.3. Comparison of GCS-R Scores between the Two Groups

The CRS-R scores in the experimental group before and after intervention were (3.54 ± 1.17) and (20.25 ± 1.37) points, respectively, and the scores in the control group were (3.59 ± 1.18) and (17.14 ± 1.26) points, respectively. The experimental group witnessed a higher GCS-R score, as compared to the control group (*P* < 0.05). See Figure 1.

RETRACTED

### 3.4. Comparison of the Nursing Effect between the Two Groups

In the experimental group, the markedly effective rate was 68.89% (31/45), the effective rate was 28.89% (13/45), the invalid rate was 2.22% (1/45), and the total effective rate was 97.78% (44/45); In the control group, the markedly effective rate was 51.11% (21/45), the effective rate was 35.56% (16/45), the invalid rate was 17.78% (8/45), and the total effective rate was 82.22% (37/45). The experimental group yielded a more favorable outcome in terms of the nursing effect (*P* < 0.05), as shown in Figure 2.

### 3.5. Comparison of GQOLI-74 Scores between the Two Groups

In comparison with the control group, results in Figure 3 presented a superior level of GQOLI-74 score in the experimental group (*P* < 0.05). The abscissa represented before and after intervention, and the ordinate represented GQOLI-74 scores. The GQOLI-74 scores in the experimental group before and after intervention were (46.44 ± 7.88) and (82.33 ± 4.98) points, respectively, and the scores in the control group were (46.72 ± 7.43) and (61.25 ± 4.22) points, respectively.

### 3.6. Comparison of BI Scores between the Two Groups

The abscissa represented before and after intervention, and the ordinate represented BI scores. The BI scores in the experimental group before and after intervention were (51.24 ± 2.34) and (88.25 ± 1.27) points, respectively, and the BI scores in the control group were (50.89 ± 2.56) and (69.77 ± 1.25) points, respectively. A superior level of the BI score of the experimental group was obtained compared with the control group (*P* < 0.05). See Figure 4.

### 3.7. Comparison of the Incidence of Complications between the Two Groups

In the experimental group, there were 0 (0.00%) intracranial infections, 1 (2.22%) stress injury, and 0 (0.00%) pulmonary infections, for an overall complication rate of 2.22%; in the control group, there was 1 (2.22%) intracranial infection, 6 (13.33%) stress injuries, and 5 (11.11%) pulmonary infections, for an overall complication rate of 26.67%. The overall complication rate was 26.67%. The experimental group showed a lower incidence of complications, as compared to the control group (*P* < 0.05), as shown in Table 3.

## 4. Discussion

Aneurysmal subarachnoid hemorrhage is classified as a critical disease with a high disability and fatality rate. Aneurysmal subarachnoid hemorrhage should generally require surgical removal of blood from the subarachnoid space and surgical removal of the aneurysm [21]. If the hemorrhage is more than 20 ml, the blood must be removed from the brain tissue to prevent pressure on the brain, especially if there is an aneurysm, to prevent re-rupture and cerebral hemorrhage [22]. At present, surgery is mainly used for treatment in clinical practice, which drives down the disability and fatality rate but tends to cause postoperative coma. As the patient's brain tissue and cranial nerves have been damaged, it is necessary to repair the damaged nerve cells, re-establish nerve function, and promote the patient's recovery. Conventional care is now the usual clinical choice to restore consciousness, but with less than satisfactory results [23–26].

RETRACTED

The whole-course responsibility nursing can effectively alleviate the workload of nursing staff, and it has substantially changed the traditional nursing model. In the whole process of responsible nursing, nursing meetings should be held regularly to analyze the problems existing in the nursing process and pay close attention to the changes of the patient's condition. High-quality nursing is a patient-centered approach to nursing, which requires the development of appropriate nursing measures according to the patient's condition and the maintenance of a comfortable treatment environment. The tactile arousal intervention used in this study is a novel form of arousal. The principle of tactile arousal intervention is that extraperitoneal stimulation acts on the damaged brain tissue of patients, thereby promoting new neural pathways, helping patients establish new connections between neurons and synapses, repairing nerve function, promoting blood circulation, and restoring patients. Consciousness. Auditory wake-up intervention is also a new type of arousal. The main principle is to provide information coding for patients by calling to form stimulation, to stimulate the body's reflex mechanism, help patients form memory traces, and then promote membrane potential to produce action potential [27–29]. For patients with severe aneurysmal subarachnoid hemorrhage and postoperative coma, the application of whole-course responsibility nursing combined with high-quality nursing intervention can effectively improve the excitability of the patient's cerebral cortex. Tactile and auditory arousal can help to wake up the function of the cerebral cortex, restore the function of brain tissue, and substantially shorten the awakening time of patients. As severe aneurysmal subarachnoid hemorrhage patients with postoperative coma require a long-term in-bed period, they are highly susceptible to pressure injuries and pulmonary infections. Results of the study highlighted that the GCS score of the experimental group was higher (*P* < 0.05 [30], whose article pointed out that “the observation group's limb response, eye-opening response, and language response were (4.64 ± 1.09), (3.49 ± 0.56) and (4.11 ± 0.64) points, respectively, and those in the control group were (3.14 ± 0.94), (2.49 ± 0.55) and (3.11 ± 0.54) points, respectively; the observation group showed higher levels of GCS scores compared with the other group (*P* < 0.05),” indicating that compared with conventional nursing, whole-course responsibility nursing combined with high-quality nursing intervention can effectively improve patient's coma degree, help patients regain consciousness, and restore the mental state.

RETRACTED

In the treatment of subarachnoid hemorrhage in TCM, the acute phase can reduce the occurrence of cerebral oedema and avoid coma [31]. During psychiatric resuscitation, the use of TCM, acupuncture, and other conditions facilitates the recovery of neurological impairments, such as limb function and gastrointestinal function; while at the same time, it improves the patient's nutritional support, enhances immunity, and greatly assists the overall status of resuscitation [32]. Therefore, it is recommended that TCM treatment of subarachnoid hemorrhage be maintained throughout the treatment process, if necessary, to achieve better outcomes [33].

## 5. Conclusion

In conclusion, the whole-course responsibility nursing combined with high-quality nursing intervention applied to severe aneurysmal subarachnoid hemorrhage patients with postoperative coma can improve the patient's level of life and reduce the incidence of complications. It is worthy of practical application. [34].

## Figures and Tables

**Figure 1:** Comparison of GCS-R scores between the two groups ($\bar{x}$ ± *s*). The abscissa represented before and after intervention, and the ordinate represented CRS-R scores, points; The CRS-R scores in the experimental group before and after intervention were (3.54 ± 1.17) and (20.25 ± 1.37) points, respectively, and those in the control group were (3.59 ± 1.18) and (17.14 ± 1.26) points, respectively; ^*∗*^Significant difference in CRS-R score in the experimental group before and after intervention (*t* = 62.219, *P* < 0.001); ^*∗∗*^Ssignificant difference in CRS-R score in the control group before and after intervention (*t* = 52.655, *P* < 0.001); ^*∗∗∗*^Ssignificant difference in CRS-R score between the two groups (*t* = 11.208, *P* < 0.001).

**Figure 2:** Comparison of nursing effect between the two groups (*n* (%)). (a) The nursing effect in the experimental group. (b) The nursing effect in the control group. In the experimental group, the markedly effective rate was 68.89% (31/45), the effective rate was 28.89% (13/45), the invalid rate was 2.22% (1/45), and the total effective rate was 97.78% (44/45); In the control group, the markedly effective rate was 51.11% (21/45), the effective rate was 35.56% (16/45), the invalid rate was 17.78% (8/45), and the total effective rate was 82.22% (37/45). After intervention, there was significant difference between the two groups (*x*^2^ = 6.049, *P*=0.014).

RETRACTED

**Figure 3:** Comparison of GQOLI-74 scores between the two groups ($\bar{x}$ ± *s*). The abscissa represented before and after intervention, and the ordinate represented GQOLI-74 scores, points; The GQOLI-74 scores in the experimental group before and after intervention were (46.44 ± 7.88) and (82.33 ± 4.98) points, respectively, and those in the control group were (46.72 ± 7.43) and (61.25 ± 4.22) points, respectively; ^*∗*^Significant difference in GQOLI-74 score in the experimental group before and after intervention (*t* = 25.828, *P* < 0.001); ^*∗∗*^Significant difference in GQOLI-74 score in the control group before and after intervention (*t* = 11.407, *P* < 0.001); ^*∗∗∗*^Significant difference in GQOLI-74 score between the two groups (*t* = 21.663, *P* < 0.001).

**Figure 4:** Comparison of BI scores between the two groups ($\bar{x}$ ± *s*). The abscissa represented before and after intervention, and the ordinate represented BI scores, points; The BI scores in the experimental group before and after intervention were (51.24 ± 2.34) and (88.25 ± 1.27) points, respectively, and those in the control group were (50.89 ± 2.56) and (69.77 ± 1.25) points, respectively; ^*∗*^Significant difference in BI score in the experimental group before and after intervention (*t* = 93.250, *P* < 0.001); ^*∗∗*^Significant difference in BI score in the control group before and after intervention (*t* = 44.456, *P* < 0.001); ^*∗∗∗*^Significant difference in BI score between the two groups (*t* = 69.568, *P* < 0.001).

**Table 1:** Comparison of general information between the two groups (*n* (%)).

	Experimental group (*n* = 45)	Control group (*n* = 45)	*x* ^2^ or *t* value	*P*
Age (years)			0.086	0.932
	46.75 ± 3.32	46.69 ± 3.29		

*Gender*			0.178	0.673
Male	23 (51.11)	21 (46.67)		
Female	22 (48.89)	24 (53.33)		

BMI (kg/m^2^)			1.119	0.266
	26.27 ± 1.59	25.89 ± 1.63		

*Smoking*			0.045	0.832
Yes	20 (44.44)	21 (46.67)		
No	25 (55.56)	24 (53.33)		

*Drinking*			0.178	0.673
Yes	22 (48.89)	24 (53.33)		
No	23 (51.11)	21 (46.67)		

*Place of residence*			0.050	0.822
Urban	31 (68.89)	30 (66.67)		
Rural	14 (31.11)	15 (33.33)		

**Table 2:** Comparison of GCS scores between the two groups (*x* ± *s*).

Group	No.	Limb response		Eye-opening response		Language response	
		Before intervention	After intervention	Before intervention	After intervention	Before intervention	After intervention
Experimental group	45	2.31 ± 0.47	4.73 ± 1.12	1.96 ± 0.24	3.51 ± 0.49	2.23 ± 0.76	4.13 ± 0.67
Control group	45	2.46 ± 0.42	3.17 ± 0.93	1.83 ± 0.37	2.18 ± 0.54	2.29 ± 0.77	3.12 ± 0.47
*t* value		1.596	7.188	1.977	12.236	0.372	8.279
*P*		0.114	<0.001	0.051	<0.001	0.711	<0.001

RETRACTED

**Table 3:** Comparison of the incidence of complications between the two groups (*n* (%)).

Group	No.	Intracranial infection	Stress injury	Pulmonary infection	Incidence of complications
Experimental group	45	0 (0.00)	1 (2.22)	0 (0.00)	1 (2.22)
Control group	45	1 (2.22)	6 (13.33)	5 (11.11)	12 (26.67)
*X* ^2^ value					10.879
*P*					0.001

## Data Availability

The datasets used during the present study are available from the corresponding author upon reasonable request.
